# A Comparative Study of Cultural and Traditional Education in Primary and Secondary Schools in Developed Countries Based on the MOPSO-CD-DNN Model

**DOI:** 10.1155/2022/3973763

**Published:** 2022-07-12

**Authors:** Chunsen Hu

**Affiliations:** Hubei Business College, Wuhan 430070, Hubei, China

## Abstract

In today's globalization, cultural and traditional education in primary and secondary schools has become the core of a country's future development, and how to improve the educational effect of cultural and traditional education in primary and secondary schools and find the development direction of cultural and traditional education has become the top priority. In response to this problem, this study proposes a MOPSO-CD-DNN hybrid prediction model, which introduces an optimization algorithm to optimize the parameters of the deep learning model. In this study, multiple benchmark models and evaluation methods are used for comparative research. The results show that the MOPSO-CD-DNN model has significant advantages in both prediction accuracy and prediction stability. Compared with other models, the prediction accuracy *G* value (average) is improved by 4.66%, 7.43%, and 9.25%, and the standard deviation (*G* value) is decreased by 0.001, 0.0502, and 0.0413, indicating its effectiveness and applicability to cultural tradition education. In addition, the introduction of the multiobjective optimization algorithm significantly improves the generalization ability of the model, and the prediction effect is significantly better than the single-objective optimization algorithm.

## 1. Introduction

Cultural tradition is the cultural spirit that originated from the life and practice of past dynasties and continues to this day in the process of continuous renewal and development [1]. It arises from the past but also exists in the present. As an organized social activity, education can be said to be a cultural phenomenon, the basic form of cultural inheritance and innovation, and the embodiment of the cultural function of education [2]. In the era of globalization, how does education cultivate modern citizens with the spirit of national culture, so that the national cultural tradition can be inherited and the national cultural literacy can be improved. For this issue, we need to broaden our horizons and effectively learn from the educational experience of other countries [3]. Therefore, this paper takes Japan and Singapore as the research objects and deeply analyzes how the two countries cultivate modern citizens who are condensed by cultural traditions through the education of cultural traditions in primary and secondary schools. [4, 5] Therefore, it is extremely necessary to study cultural tradition education.

Some scholars have analyzed [6, 7] the characteristics of school moral education in Japan and Singapore at the level of cultural traditions. The main manifestations are as follows: first, as an oriental cultural tradition, and influenced by Confucianism, moral education is placed in the first place. First place is in school education. Secondly, in the collision and exchange of Eastern and Western cultures, the reasonable elements of Western educational values are drawn to reconstruct the common values of the nation. Moral education not only adapts to national traditions but also integrates Eastern and Western cultural strengths. Third, pay attention to the comprehensive cultivation of people's quality, develop modern content and modern methods, and reflect the coordination in the conflict between traditional spirit and modern consciousness. Some scholars have done a comparative study on moral education in Japan and Singapore and made a comparison on the basis of analyzing the goals and contents of moral education in Japan and Singapore. The difference is that Japan cultivates perfect personality and emphasizes the formation of the “Yawa soul” [8]; Singapore, because of the historical background of immigrant society and cultural diversity, aims to cultivate “Singaporeans,” aiming to achieve the independence and development of a newly established country [9]. The similarities are that they have absorbed the essence of Eastern and Western cultures, and moral education ideas all emphasize loyalty to the country and serve the country [10]. Other scholars have analyzed the characteristics of ideological and political education in Japan and Singapore, which are as follows: advocating common values and enhancing the sense of identity [11]; cherishing and inheriting traditions, highlighting nationality [12]; comprehensive school, family, and society Collaboration; eclectic, integration of East and West; implement ideological and political education with moral courses as the main way, and other courses and activities also tap moral education factors [13]. Some scholars have made a different analysis of moral education in Japanese and Singaporean schools. In terms of guiding ideology, Japan is controlled by neoconservatism and neoliberalism, while Singapore is deeply influenced by Confucian ethics [14]; in terms of mainstream values, Japan cultivates the utilitarian values of “obedient and participatory” citizens, while Singapore pays attention to implementing I am a Singaporean common value [15]; in terms of methods, Japan pays attention to moral reasoning, while Singapore pays attention to moral practice; in the moral education environment, Japan supports the impoverishment of the life and culture of moral education, while Singapore emphasizes family, social moral education environment, and school moral education combined with [16]. In recent years, with the continuous development of deep learning technology, it has been widely used in various fields. The advantage of deep learning is that it learns step by step through multiple networks, extracts complex and effective features, and has higher prediction accuracy and generalization ability. Some researchers have used deep neural networks to predict the development of cultural education. The experimental results show that DNN has good prediction potential for time series [17]. Some researchers have found that the LSTM neural network can effectively capture the changes in time series in the study of the cultural comparison research of different countries [18]. At present, there are few studies on the application of deep learning in cultural and traditional education in primary and secondary schools. At the same time, it should be noted that the choice of parameters will also have an important impact on the prediction effect of the model [19]. At present, the optimization methods for model parameters mainly include cross-validation, grid search, and intelligent optimization algorithms. Some researchers [20] used the CSA algorithm to optimize the weights of the feedforward neural network, and the results showed that the prediction effect of the model was significantly improved, reaching 90.30%.

The above studies generally use a single-objective optimization method, but the prediction of cultural and traditional education is affected by many factors, not only the prediction accuracy but also the model stability should be considered. Zhang et al. [21] introduced the NSGA-III multiobjective algorithm to forecast the power load, and the results showed that the prediction performance of the NSGA-III optimized model was significantly better than that of the single-objective model. Representative multiobjective optimization algorithms mainly include PAES, SPEA2, and NSGA-II. Among them, MOPSO is a multiobjective optimization algorithm based on Pareto domination and external archiving mechanism, which has the advantages of good convergence characteristics and low time complexity. In a comparative study with other multiobjective optimization algorithms, it was found that MOPSO significantly outperformed methods such as NSGA-II, PAES, and micro DE [22]. To sum up, this paper combines MOPSO-CD and DNN to construct a comparative prediction model of cultural and traditional education in primary and secondary schools in developed countries, hoping to learn from the current cultural and traditional education in my country, so as to infiltrate cultural traditions into school education. In goal construction, curriculum construction, and teaching design, let cultural tradition education become an organic component of the school education system and cultivate primary and secondary school students who can inherit and carry forward Chinese cultural traditions and have cultural awareness and cultural spiritual heritage.

## 2. Building a Predictive Model

### 2.1. DNN Model

Deep learning has been widely used in the fields of text detection, speech, and face recognition, and natural language processing and achieved excellent results [23]. Compared with the traditional shallow machine learning method, it has the advantages of strong feature extraction ability, simple model structure, low training difficulty, and fast convergence speed. Compared with the traditional neural network, the deep neural network (DNN) inherits the structure of the traditional neural network; that is, it has a three-layer network (see Figure 1), in which the hidden layer reaches more than 6 layers [24].

In Figure 1, the DNN network structure layer can be mainly divided into three layers, the first layer is the input layer, the second layer is the hidden layer, and the third layer is the output layer, in which the layers are fully connected; that is, the first layer of any neuron in the *n* layer must be connected with any neuron in the *n* + 1th layer, and the connection relationship can be expressed by the formula (1), and the formula (2) is the basic model form of the deep neural network.

(1) $$\begin{array}{c} s=\sum_{i=1}^{n}w_{i}x_{i}+b, \end{array}$$

(2) $$\begin{array}{c} y_{m}=f\left(\sum_{i=1}^{n}w_{\text{im}}x_{i}+b_{m}\right), \end{array}$$

where *w* is the weight, *b* is the bias, *x*_*i*_ is the neural unit, and *f*(*·*) is the activation function. Common activation functions include sigmoid function and tanh function. Sigmoid functions are nonlinear functions. When the input data are small, the output is close to 0; as the input increases, the output is close to 1. *tanh* is a symmetric function centered at zero, and its model training process converges faster than the sigmoid function. This paper first selects appropriate samples and input features based on the characteristics and requirements of the comparison of traditional culture and education in primary and secondary schools in different developed countries, then trains the model, determines the relevant parameters of the deep network model, and selects an appropriate prediction model; finally, the test sample data are used. The predictive ability of the model is tested.

### 2.2. MOPSO Model

All particles fly at a certain speed in the search space and find the global optimal value through the currently searched optimal value. Particle swarm optimization is an iterative-based optimization algorithm. The system is initialized to a set of random solutions, and the optimal value is found through iteration. It is one of the generalized swarm intelligence methods for solving optimization nonlinear problems. The swarm search algorithm and the particle swarm algorithm have few parameters, and it is easy to fall into the problem of local optimality while the multiobjective particle swarm can be used to optimize more than one target parameter, and there are contradictions between the objectives, and there is no uniform measurement standard, and in the case of the unit of measurement, it is an optimization algorithm that can obtain a uniformly distributed noninferior solution set covering the entire search space with as little computing resources as possible.

When using the MOPSO algorithm to achieve target optimization, a set of random solutions (called “particles”) will be obtained first, and each particle will have a specific location and initial velocity associated with it *V*_*i*_. At the same time, according to the fitness determined by the objective function, the optimal position pid and the current position *X*_*i*_ under the current search progress will be determined. At the same time, each particle can obtain the optimal position pgd of the entire population. Therefore, the MOPSO algorithm can be regarded as a self-organizing behavior in which each particle transmits information in a certain space according to a certain rule or method and continuously corrects itself according to the deviation between the actual position and the optimal position.

### 2.3. MOPSO-CD Model

Multiobjective particle swarm optimization based on crowding distance (MOPSO-CD) is a heuristic evolutionary multiobjective optimization algorithm [25]. As a derivative model of MOPSO, its main idea is to use the strategy of archiving and retaining the elite solution, using the random selection method to select the elite from the external archive set as the global optimal solution of the particle, and at the same time introducing the dynamic nonuniform mutation operator, and finally, the goal of maintaining the diversity of particles, slowing down the convergence speed of the algorithm, and avoiding premature convergence is achieved. Studies have shown that this method is more efficient and practical than the classical method [26].

### 2.4. MOPSO-CD-DNN Hybrid Prediction Model

This paper uses the multiobjective particle swarm optimization algorithm based on crowding distance (MOPSO-CD) to optimize the parameters of DNN, analyzes the comparison of cultural and traditional education in primary and secondary schools in developed countries, and then predicts the cultural and traditional education of Chinese primary and secondary schools. The specific implementation process of the model is as follows:

  Step 1: *Data selection and preprocessing*. This paper selects the experimental sample set according to the target principle of the same industry in the same period and selects the traditional culture education of Japan and Singapore as the main sample, and the rest as the positive sample. Then, the relevant data are standardized (Z-score) to eliminate the influence of the index dimension, and PCA is used to extract factors, and after eliminating redundant characteristic variables, a cultural education prediction model is constructed. In addition, in the data sample division, the training set (70%) and the test set (30%) are randomly selected.
  Step 2: *Model training and parameter optimization*. Using the training set data set, a deep learning model is used to train a cultural and educational development prediction model. At the same time, the MOPSO-CD algorithm is used to optimize the selection of DNN parameters. The optimized parameters are used to predict the cultural and educational situation of primary and secondary schools on the test set. Among them, the objective functions of the MOPSO-CD optimization algorithm are TPR, TNR, EPR, and ENR, with a total of 4 objective functions.
  Step 3: *Model testing*. The trained MOPSO-CD-DNN traditional culture education prediction model for primary and secondary schools is tested on the test set, and the corresponding experimental results are obtained to verify the performance of the cultural development prediction model proposed in this paper.
  Step 4: *Evaluation of traditional cultural education mixed prediction model*. A variety of model performance evaluation indicators are used to test the MOPSO-CD-DNN mixed traditional culture education prediction model. In addition, this paper uses three comparative studies to further examine the effectiveness and advancement of the MOPSO-CD-DNN model. First, through the comparison and selection of single models such as SVM and BPNN, the superiority of using the DNN model in the hybrid early warning model is demonstrated. Second, the applicability of the MOPSO-CD algorithm is verified by comparing the proposed hybrid early warning model with models such as NSGA-II-DNN. Third, the MOPSO-CD-DNN model proposed in this paper is compared with the SA-DNN and DE-DNN models, and the advantages of the multiobjective optimization algorithm in optimization efficiency and effect are investigated.

### 2.5. Evaluation of Traditional Culture Education Prediction Model

This paper uses the traditional classification accuracy to analyze the classification accuracy of the traditional cultural education prediction model and uses the evaluation index for unbalanced samples to evaluate the prediction accuracy of the traditional cultural education prediction model. The classification accuracy is the proportion of positive and negative samples that are correctly predicted to the number of positive and negative samples (TPR and TNR) and the overall accuracy (TR) [27]. The evaluation indicators for the classification of unbalanced samples are the geometric mean accuracy rate *G* and the minority class sample metric *F*. The geometric average accuracy *G* comprehensively examines the prediction performance of the model for two types of samples. If *G* is larger, it means that the model has higher accuracy in predicting both types of samples. Otherwise, the model accuracy is smaller. If *F* is larger, it means that the prediction performance of the model for traditional cultural education prediction samples is superior; otherwise, the prediction performance is worse [28]. The calculation formula of the evaluation index is as follows:

(3) $$\begin{array}{c} \text{TPR}=\frac{\text{TP}}{\text{TP}+\text{FP}}\text{,}\\ \text{TNR}=\frac{\text{TN}}{\text{TN}+\text{FN}},\\ \text{TR}=\frac{\text{TP}+\text{TN}}{\text{TP}+\text{FP}+\text{TN}+\text{FN}}\text{,}\\ G=\sqrt{\frac{\text{TN}}{\text{TN}+\text{FN}}\times \frac{\text{TP}}{\text{FP}+\text{TP}}},\\ F=\frac{2\times \text{TN}/\text{TN}+\text{FN}\times \text{TN}/\text{TN}+\text{FP}}{\text{TN}/\text{TN}+\text{FN}+\text{TN}/\text{TN}+\text{FP}}. \end{array}$$

### 2.6. Selection of Characteristic Indicators

Since there is no recognized standard for the characteristic indicators used in the traditional cultural education forecasting model, this paper draws on the relevant research to select the characteristic indicators and initially obtains the traditional cultural education forecasting system. Finally, four key indicators of survival, efficiency, ability, and value are selected as the input features of the MOPSO-CDD-DNN mixed traditional culture education prediction model [29]. In this paper, the above indicators are selected to construct a feature indicator set, and the PCA method is used to reduce the dimensionality of the indicators. Before performing PCA, KMO test and Bartlett sphericity test should be performed on the characteristic indicators to judge whether each standard is suitable for principal component analysis.

## 3. Comparison of Predictive Performance between Traditional Cultural Education Model and Other Models

### 3.1. Prediction Accuracy Comparison

In order to evaluate the traditional cultural education prediction model more comprehensively, in addition to the overall accuracy of TR, this paper also gives the prediction accuracy (TPR and TNR) of positive samples and negative samples. Based on the results in Table 1, the MOPSO-CD-DNN model constructed in this paper has the best prediction accuracy, which is about 4 percentage points behind the second best model NSGA-II-DNN in TR. Its evaluation indicators TPR, TNR, and TR are 72.88%, 75.56%, and 74.04%, respectively, which are higher than the other six prediction models, indicating that the MOPSO-CD-DNN method has better performance in enterprise financial risk prediction. In addition, the prediction performance of NSGA-II-DNN and MOPSO-CD-DNN is better, indicating that the multiobjective optimization algorithm is better than the single-objective method in prediction effect.

The above experimental results only analyze the differences of the models from the numerical value of the prediction accuracy but lack the significance of mathematical statistics. Therefore, in order to strengthen the scientificity and objectivity of the obtained results, on the basis of the results in Table 1, the paired-sample *t*-test and Friedman test were used to test the significance of the prediction results to judge whether there was a significant difference in the prediction performance of different models. The specific experimental results are shown in Tables 2 and 3.

The results in Table 2 show that, except that the paired-sample *t*-tests on TNR for MOPSO-CD-DNN and NSGA-II-DNN were significant at the 5% level, the *T*-tests of the remaining models and MOPSO-CD-DNN on each indicator reject the null hypothesis at the 1% significance level, indicating that the MOPSO-CD-DNN model has significant differences in TPR, TNR, and TR compared with other models, its traditional cultural education prediction effect is better. In addition, it can be found from Table 3 that the *F* and *P* values of TPR are 26.657 and 0.001, respectively, while the *F* values of TNR and TR are 27.771 and 26.225, respectively.

### 3.2. Predictive Stability Comparison

Since paired sampling in a 1 : 1 ratio will have a certain impact on the randomness of the sample, and in order to compare the prediction stability of the MOPSO-CD-DNN model with the NSGA-II-DNN, DE-DNN, and SA-DNN models, therefore, this paper examines the robustness of the MOPSO-CD-DNN traditional culture and education prediction model by increasing the number of positive samples paired with negative samples and changing the ratio between positive and negative samples. Specifically, firstly, the ratio between the traditional culture education sample and the normal sample is set to 1 : 2, 1 : 3, 1 : 4, 1 : 5, and 1 : 6, totaling five. Then, the changes in the prediction accuracy of the four types of models under these five proportions are analyzed, so as to judge the prediction stability of the MOPSO-CD-DNN model. Since the samples under the five proportions are no longer balanced samples, it is necessary to introduce metrics specifically for unbalanced samples to evaluate the predictive performance of the model. The results of the model experiment are shown in Figure 2.

As can be seen from the above figure, under different proportions of positive and negative samples, the *G* value (0.7803) of the MOPSO-CD-DNN model is higher than other models, and the *F* value is poor, but its *F* mean (0.5902) is higher than other models with the smallest standard deviation. It shows that the NSGA-II-DNN, DE-DNN, and SA-DNN models are inferior to MOPSO-CD-DNN for both traditional culture education samples and nontraditional culture education samples. From the graph in Figure 2, the prediction accuracy *G* and *F* of the MOPSO-CD-DNN model are relatively more stable and less volatile, and the standard deviations of *G* and *F* are 0.0097 and 0.0462, respectively, which are also significantly lower than other methods. This shows that the prediction results of the two types of samples are stable under different proportions of traditional cultural education samples.

### 3.3. Sensitivity Analysis of MOPSO-CD Algorithm

The MOPSO-CD multiobjective optimization algorithm contains three main parameters: the number of particle swarms (popsize), the number of iterations (generations), and the archive size (archivesize), which can significantly affect the effectiveness of the proposed hybrid model for traditional culture and education prediction. Appropriate parameters will improve forecast accuracy and forecast efficiency. Therefore, it is necessary to explore the influence of the parameter changes of the MOPSO-CD model on the prediction performance of traditional culture education by modifying one of the three parameters and keeping the other parameters unchanged (see Table 4).

Table 4 shows that changes in the number of particle swarms, the number of iterations, and the file size have a significant impact on the prediction performance of MOPSO-CD-DNN. For example, with the increase in the number of iterations, TR shows a law of first increasing and then decreasing. When the number of iterations is 8, TR reaches the maximum value (74.04%), and after that, TR gradually decreases. Therefore, changes in the number of iterations will affect the predictive ability of the proposed traditional cultural and educational hybrid prediction model. The changes in MOPSO-CD parameters will obviously affect the prediction effect of the traditional cultural education mixed prediction model. Inappropriate and poor parameters will lead to the failure to find the optimal initial parameters of the DNN, thus reducing the predictive ability of the MOPSO-CD-DNN hybrid model. According to the experimental results, this paper sets the number of particle swarms to 100, the number of iterations to 8, and the file size to 250.

## 4. Conclusion

Traditional culture education in primary and secondary schools has always been one of the hotspots in the education sector. This paper fully considers the complexity of traditional culture education forecasting. Singapore and Japan are compared as developed countries. By combining multiobjective optimization algorithm and deep learning technology, a traditional culture education prediction method based on MOPSO-CD is constructed, and it is successfully used in traditional culture education prediction, and compared with other 6 benchmark models. The results show that (1) in terms of prediction accuracy, the MOPSO-CD-DNN method has better prediction ability, and its prediction accuracy is statistically significant compared with other methods; (2) in terms of prediction robustness, MOPSO-CD-DNN can effectively control the fluctuation degree of prediction accuracy and improve the stability of prediction. Compared with NSGA-II-DNN, DE-DNN, and SA-DNN, the prediction accuracy is improved. The *G* value (mean value) increased by 4.66%, 7.43%, and 9.25%, and the standard deviation (G value) decreased by 0.001, 0.0502, and 0.0413; (3) the introduction of multiobjective optimization algorithm can effectively enhance the prediction ability and generalization ability of DNN, avoid the shortcomings of single-objective optimization, and improve the learning ability for unbalanced samples.

## Figures and Tables

**Figure 1:** Traditional BP neural network and deep neural network structure diagram.

**Figure 2:** Comparison of the prediction results of the four types of models under different sample proportions. (a) *F* value, (b) *G* value.

**Table 1:** Comparison of the classification results of each model.

Model	TPR/%	TNR/%	TR/%
BPNN	57.81	57.50	57.69
SVM	65.79	56.06	59.61
DNN	60.00	59.09	59.62
DE-DNN	64.15	60.78	62.50
SA-DNN	66.67	62.26	64.42
NSGA-II-DNN	68.85	72.09	70.19
MOPSO-CD-DNN	72.88	75.56	74.04

**Table 2:** Paired-sample *t*-test for prediction accuracy of each model.

Model	MOPSO-CD-DNN		
	TPR/%	TNR/%	TR/%
NSGA-II-DNN	4.926^*∗∗∗*^	3.336^*∗∗*^	7.202^*∗∗∗*^
SA-DNN	12.341^*∗∗∗*^	8.214^*∗∗∗*^	20.396^*∗∗∗*^
DE-DNN	13.046^*∗∗∗*^	8.647^*∗∗∗*^	17.393^*∗∗∗*^
DNN	9.168^*∗∗∗*^	8.810^*∗∗∗*^	10.525^*∗∗∗*^
SVM	6.182^*∗∗∗*^	33.698^*∗∗∗*^	18.779^*∗∗∗*^
BPNN	23.877^*∗∗∗*^	24.342^*∗∗∗*^	32.163^*∗∗∗*^

*Note.* ^*∗*^means *p* < 0.1, ^*∗∗*^means *p* < 0.05, ^*∗∗∗*^means *p* < 0.01.

**Table 3:** *F* test of prediction accuracy of each model.

	Compare models	TPR/%	TNR/%	TR/%
MOPSO-CD-DNN	NSGA-II-DNN	*F* = 26.657 *P*=0.001	*F* = 27.771 *P*=0.001	*F* = 26.225 *P*=0.001
	SA-DNN			
	DE-DNN			
	DNN			
	SVM			
	BPNN			

*Note.* ^*∗*^means *p* < 0.1, ^*∗∗*^means *p* < 0.05, ^*∗∗∗*^means *p* < 0.01.

**Table 4:** Sensitivity analysis results of MOPSO-CD algorithm.

Parameter	Parameter value	TPR/%	TNR/%	TR/%
Number of particle swarms	50	67.92	64.71	66.35
	100	72.88	75.56	74.04
	150	68.97	69.57	69.23
	200	74.47	66.67	70.19
	250	68.42	68.09	68.27
	300	68.25	73.17	70.19

Number of iterations	58	73.91	65.52	69.23
	15	72.88	75.56	74.04
	23	66.18	75.00	69.23
	35	65.28	78.13	69.23
	50	69.23	65.38	67.31
	130	68.52	66.00	67.31

File size	160	71.11	62.71	66.35
	190	71.69	68.63	70.19
	220	70.83	64.29	67.31
	250	67.24	67.39	67.31
	280	72.88	75.56	74.04
	50	68.42	68.09	68.27

## Data Availability

The dataset can be accessed upon request.
